This article has been retracted.

# Neuronal Apoptosis in Patients with Liver Cirrhosis and Neuronal Epileptiform Discharge Model Based upon Multi-Modal Fusion Deep Learning

**DOI:** 10.1155/2022/2203737

**Published:** 2022-03-17

**Authors:** Nannan Chi, Xiuping Wang, Yun Yu, Manman Wu, Jianan Yu

**Affiliations:** ^1^Digestive Department, the First Affiliated Hospital of Jiamusi University, Jiamusi 154000, Heilongjiang, China; ^2^Department of Neurology, the First Affiliated Hospital of Jiamusi University, Jiamusi 154000, Heilongjiang, China; ^3^3 Medical Education Department, the First Affiliated Hospital of Jiamusi University, Jiamusi 154000, Heilongjiang, China; ^4^Graduate Department, Jiamusi University, Jiamusi 154000, Heilongjiang, China

## Abstract

Neurons refer to nerve cells. Each neuron is connected with thousands of other neurons to form a corresponding functional area and carry out complex communication with other functional areas. Its importance to the human body is self-evident. There are also many scholars studying the mechanism of apoptosis. This paper proposes a study of neuronal apoptosis in patients with liver cirrhosis and neuronal epileptiform discharge models based on multi-modal fusion deep learning, aiming to study the influencing factors of abnormal neuronal discharge in the brain. The method in this paper is to study multi-modal information fusion methods, perform Bayesian inference, and analyze multi-modal medical data. The function of these research methods is to obtain the relationship between the independence of information and the intersection of information among modalities. In the neuronal epileptiform discharge model, the mRNA expression level of the necroptotic signaling pathway related protein was detected, and the mechanism of neuronal necrosis in patients with liver cirrhosis was explored. Experiments show that the neuron recognition rate has been increased from 67.2% to 84.5%, and the time has been reduced, proving the effectiveness of deep learning.

## 1. Introduction

### 1.1. Background

In medical imaging, the use of deep learning for automatic diagnosis has become an unstoppable power [1, 2]. However, it is limited by factors such as data acquisition channels, and most of the existing researches focus on single-modality images. However, single-modal images are often very limited in the expression of pathological information. Therefore, it is very necessary to obtain more comprehensive pathological information by studying the image data of multiple modalities. Addressing the issue of the single-modal interaction being very much affected by user operations and the interaction efficiency being low, this paper constructs the fusion of gestures, voice, sensor information, and intelligent interaction methods at the decision-making level. Furthermore, this paper proposes an intelligent navigation interaction model oriented to multi-modal fusion. First of all, this paper establishes three modal information data sets and intention analysis to construct multi-modal information intersection and information independent functions. Next, based on the directed graph, this paper proposes an interaction strategy to realize the understanding of the user's intention of multi-modal information fusion. Finally, this paper proposes a navigation interaction mode based on multi-modal intention understanding. It can correctly guide the user's operation behavior and solve the problem of difficult operation.

### 1.2. Significance

The purpose of this research and application was to provide better medical resources for small and medium medical institutions. It is of great significance for telemedicine and medical care where education and experimental conditions are obviously lacking [3, 4]. In the first homogenous multimodal image for the liver cirrhosis grading task, this paper employs histogram equalization technique to enhance image detail and contrast. It optimizes the enhancement of liver cirrhosis, and has better classification indicators than previous methods. In the second heterogeneous ultrasound and electronic medical record for the early diagnosis of cardiovascular disease, in view of various factors such as data acquisition channels, the research of multi-modal ultrasound imaging is rarely involved, and ultrasound imaging has an irreplaceable role for special populations. This article uses the fusion method of homogenous multi-modal imaging and heterogeneous electronic medical records for hospital data for practical project applications. And, this article has carried on the visual explanation analysis to the training process of the homology multi-modal ultrasound image fusion. It has a strong practical guiding significance.

### 1.3. Related Work

For the neuron epileptiform discharge model, many scholars have carried out research on it. With the recent resurgence of neural networks and the proliferation of large amounts of unlabeled multi-modal data, Vukoti V believes that recommendation systems and multi-modal retrieval systems based on continuous representation spaces and deep learning methods are becoming more and more concerned. He introduced an alternative to advanced multi-modal fusion. The cross-modal conversion is realized by projecting the symmetrical encoder onto the bidirectional deep neural network [5]. Luo proposed a new multi-modal medical image fusion method based on environmental information. The experimental result is that compared with some typical fusion methods, the fusion method he proposed can effectively suppress color distortion and provide better fusion quality [6]. LiS proposes a point-to-point convolutional network called attention-based multi-modal fusion network, which is used to infer the task completion status of a 3D scene from a single-view RGB. Compared with the previous method that only used the extraction of semantic features from RGB-D images, the method he proposed uses the experience of inferring semantic segmentation from RGB-D images. The results show that his method achieves gains of 2.5% and 2.6% on the synthetic SUNCG-RGBD data set NYUv2 data set, respectively [7]. Kumthekar A proposed a technology based on deep learning technology for automatic cloud detection in multispectral images. These different initial layers are designed to increase the width of the network by replacing the standard convolutional layer. They extract multi-scale features without loss of resolution and maintain the same output size as the input image size. Reducing the computational complexity by reducing the number of parameters, using fewer spectral bands and deconvolution [8]. The classification accuracy of the model developed by Zhang differs significantly when applied to an independent test data set. He explored two potential training strategies to solve the over-fitting problem in AF detection [9]. Liu proposed a multi-task deep learning method, which may exist in the open world of unknown classes for simultaneous classification and reconstruction. He compared the reconstructed data with the original data. Due to the lack of labels, the data is not well represented in the underlying features. He proposed two strategies based on extreme value theory, which are used in few-shot and multi-shot scenes respectively [10]. Demianenko believes that the synchronous burst firing of neuron action is a typical manifestation of brain epileptiform activity, and this firing is reflected in the EEG as a burst seizure [11]. The purpose of Zhang is to study the regulatory effect of LIUS on epileptiform discharges in mouse hippocampal slices and its underlying mechanism. The results showed that LIUS suppressed the amplitude, rate and duration of the discharge. For interictal discharge, LIUS inhibits the spontaneous spike activity of mouse pyramidal neurons and eliminates epileptiform resistance [12].

### 1.4. Innovation

In this thesis, the Li-Pilo continuous high-frequency induced epileptiform discharge model and the primary culture hippocampal neuron spontaneous repetitive epileptiform discharge model induced by magnesium-free external fluid were used in this thesis. This article uses behavioral analysis and a number of molecular biology research methods to study the effect of MK2206 on the AKT/NF-KB signaling pathway and hippocampal neuron necrosis. This article proposes some practical applications of trained models, which have excellent reference value in medical diagnosis. (1) Images of different modalities adopt a unified feature extraction method. It can be seen from the visualization data of the early diagnosis task of cardiovascular disease that the experiment did not make full use of the motion wave group modal image and the Doppler spectrum image. (2) At the feature fusion level, this instrument performed a simple splicing operation. This paper does not carry out correlation analysis on the extracted features of different modalities, and explore the potential connections between them.

## 2. Research Methods of Neuronal Apoptosis

### 2.1. Multimodal Information Fusion Method

Modality is a subdivision concept of media. Each source of information and different manifestations can be called a modality. Multi-modality in this article refers to the existence of multiple media forms for the description of the same object. According to the data media form and source of the description object, this article can divide the modalities into homogenous modalities and heterogeneous modalities. For example, images, texts, and electrical signals belong to heterogeneous multi-modality. The different sequence images produced by the same magnetic resonance equipment or the different description images produced by the same color ultrasound equipment are all homologous multi-modality [13].

By analyzing the user's possible intentions during operation, this article will obtain the relationship between information independence and the intersection of information and modalities. Therefore, this paper establishes the multi-modal information intersection function and information independent function. First, recognition is performed based on various modal inputs such as sensor information, gesture information, and voice information recognition. Then, based on the recognition result, it is determined whether it is an information cross function or an information independent function [14]. When the user's behavior status is set to Taks_*T* ∈ {*T*1, *T*2,…*Tn*}, the information cross function *F*1(Taks_*T*, *M*) is:

(1) $$\begin{array}{c} F_{1}\left({\text{Taks}}_{T},M\right)=\left\{\begin{array}{c} \begin{array}{c} T1\left(t_{1}\cap a_{4}\cap v_{1}\right)\neq \emptyset \\ \text{or}\\ t_{1}\cap a_{4}\neq a_{4}\cap v_{1}\neq \emptyset , \end{array}\\ T2\left(t_{9}\cap a_{8}\right),\\ T3\left(t_{10}\cap a_{9}\right),\\ \begin{array}{c} T4\left(t_{5}\cup a_{1}\neq \emptyset \right)\\ \text{or}\\ \left(t_{7}\cup a_{1}\right)\neq \emptyset , \end{array}\\ T5\left(t_{11}\cap a_{6}\neq \emptyset \right),\\ \vdots \\ Tn\left(t_{n+1}\cap a_{n+2}\neq \emptyset \right). \end{array}\right. \end{array}$$

In (1), Taks_*T* ∈ {*T*1, *T*2,…*Tn*}, the current behavior state Taks_*T* of the user is determined by judging the information merge function of different modalities. The information independent function *F*  *d*(Taks_*T*, *M*) is

(2) $$\begin{array}{c} Fd\left({\text{Taks}}_{T},M\right)=\left\{\begin{array}{cc} T13 & t_{3}\neq \emptyset ,\\ T14 & v_{3}\neq \emptyset ,\\ T15 & v_{4}\neq \emptyset ,\\ T16 & a_{3}\neq \emptyset ,\\ T17 & a_{10}\neq \emptyset . \end{array}\right. \end{array}$$

In (2), Taks_*T* ∈ {*T*13, *T*2,…*T*17}, the current behavior state Taks_*T* of the user is determined according to the information independent function. According to the multi-modal information fusion strategy, different behavior states Taks_*T* of users are judged. Determine the user's intention under the current trigger condition and establish the following rules:

(3) $$\begin{array}{c} \left\{\begin{array}{c} \text{Taks}\_T\neq \emptyset ⟶e_{17},\\ \text{Taks}\_T=\emptyset ⟶\emptyset . \end{array}\right. \end{array}$$

The main goal of canonical correlation analysis is to find linear projections of data from various data sources with the greatest correlation [15]. Canonical correlation analysis is a linear mathematical model. It is a multivariate statistical analysis method suitable for multi-source heterogeneous data, multi-view, and multi-scale analysis. Its purpose is to identify and quantify the relationship between two sets of variables, focusing on the correlation between the linear combination of one set of variables and the linear combination of another set of variables. The idea is to first solve the linear combination of the two variable sets to maximize the correlation coefficient [16]. Then, select the pair with the highest correlation coefficient from the linear combination pairs that are not related to the first selected linear combination pair, and so on. These selected linear combination pairs are called canonical variables, and their correlation coefficients are called canonical correlation coefficients. The canonical correlation coefficient measures the strength of the connection between these two sets of variables. This maximization technique aims to map the high-dimensional relationship between the two sets of variables to some typical variables [17].

Ultrasound image feature extraction model InceptionV3 is used in the experiment of this article to first divide the ultrasound image into four modal data sets with each modal as a unit. Then, train on each data set and save the best classification model. These four optimal models are the feature extraction models of four modes [18]. The feature extraction dimension of each mode is 128.

After the multi-modal feature fusion, this article chooses the XGBoost model as the classification model. XGBoost is mainly improved based on the gradient boosting decision tree, so the essence of XGBoost is still a combination of multiple regression trees, and each round of training is based on the previous generation. Assuming there are *n* samples, each independent sample is defined as xn, and the value range of *n* is (1,n). For each sample, the prediction result yn of XGBoost is equal to the superposition of the predicted values of K trees completed by the model training [19]. The formula is as follows:

(4) $$\begin{array}{c} {\hat{y}}_{n}=\sum_{k=1}^{K}f_{k}\left(x_{n}\right),\;f_{k}\in F\text{.} \end{array}$$

Among them, *f*_*k*_ represents the function of the k-th tree, and F represents the space of the tree. The objective function of the model is as follows:

(5) $$\begin{array}{c} L\left(\emptyset \right)=\sum_{n}l\left({\hat{y}}_{n},y_{n}\right)+\sum_{k}\Omega f_{k}. \end{array}$$

The optimization direction of the function is to minimize *L*(∅). Among them, the loss function *l*, the regular term ∑_*k*_Ω*f*_*k*_, and *O* represent the complexity of the tree, which can be further expressed as follows:

(6) $$\begin{array}{c} \Omega \left(f\right)=yT+\frac{1}{2\gamma }{\left\|\omega_{i}\right\|}^{2}. \end{array}$$

Among them, the number of leaf nodes is represented by *T*, and the score of the *i*-th leaf node is represented by *ω*_*i*_. Because the objective function is not convenient to optimize, the Taylor series is used to further optimize the function. The formula is as follows:

(7) $$\begin{array}{c} \omega_{n}^{*}=\frac{\sum_{n\in \text{In}}\partial l\left(y_{n},{\hat{y}}_{n}^{n-1}\right)}{\sum_{n\in \text{In}}\partial^{2}l\left(y_{n},{\hat{y}}_{n}^{n-1}\right)}+\gamma ,\\ L^{-n}\left(q\right)=\frac{-1}{2}\sum_{j=1}^{T}\left\{\frac{{\left[\sum_{n\in \text{In}}\partial l\left(y_{n},{\hat{y}}_{n}^{n-1}\right)\right]}^{2}}{\sum_{n\in \text{In}}\partial^{2}l\left(y_{n},{\hat{y}}_{n}^{n-1}\right)}\right\}+\gamma T. \end{array}$$

In practice, it is impossible to list the shapes of all trees for optimal calculation, so the tree is split and calculated to obtain the final objective function:

(8) $$\begin{array}{c} L_{\text{splot}}=\frac{1}{2\left\{{\left[\sum_{n\in I_{L}}\partial l\left(y_{n},{\hat{y}}_{n}^{n-1}\right)\right]}^{2}/\sum_{n\in I_{L}}\partial^{2}l\left(y_{n},{\hat{y}}_{n}^{n-1}\right)+\gamma \right\}}+\frac{{\left[\sum_{n\in I_{n}}\partial l\left(y_{n},{\hat{y}}_{n}^{n-1}\right)\right]}^{2}}{\sum_{n\in I_{n}}\partial^{2}l\left(y_{n},{\hat{y}}_{n}^{n-1}\right)+\gamma }-\gamma . \end{array}$$

Therefore, in order to merge the information between multiple modes in parallel with more reasonable weights, reduce the mutual cancellation of information between different modes, and improve accuracy, as it is necessary to set the initial value of the weight of each mode reasonably [20]. The experiments in this article are performed on each input data, and the accuracy of the segmentation results of each modal image is obtained by statistics. Using this as prior knowledge, this article expresses it as fusion weights to achieve better segmentation results.

Based on the characteristics of MRI images, it is determined that there are four modal images (Flair, T1, T1c, T2) that are closely related to the segmentation results. The weights of Flair modal images are set to *α*, *β*, *γ*, *θ*, respectively, as shown in Figure 1.

### 2.2. Deep Learning and Bayesian Inference

Deep learning is a type of machine learning algorithm that meets the following characteristics. Deep neural network is not a “black box model,” and its theoretical basis relies on general approximation theory and Bayesian inference [21–23]. Among them, the general approximation theory is described as follows:

Define *s* as any continuous nonlinear sigmoid function, namely,

(9) $$\begin{array}{c} \sigma \left(x\right)=\left\{\begin{array}{c} 1\;x⟶+\infty ,\\ 0\;x⟶-\infty . \end{array}\right. \end{array}$$

Define *G*(*x*) as a linear combination of *σ*, namely:

(10) $$\begin{array}{c} G\left(x\right)=\sum_{n=1}^{N}\alpha_{n}\sigma \left(y_{n}^{t}+b_{n}\right). \end{array}$$

Among them, *x* ∈ ∂^*n*^, *yn* ∈ ∂^*n*^, *α*_*n*_, *b*_*n*_ ∈ ∂. Let In denote the n-dimensional unit cube [0,1]^n^, and the continuous function space on In is denoted as C(In), then given any *f* ∈ *C*(In), ∀ò > 0, ∃G(x) satisfies:

(11) $$\begin{array}{c} \left|G\left(x\right)-f\left(x\right)\right|<\text{ ò},\;x\in \text{In}. \end{array}$$

The Bayesian inference theory is described as follows: The prior distribution *p*(*θ*|*α*), which is usually not easy to observe. The sample distribution *p*(X|*θ*) is also called the likelihood function, which can be considered as the marginal likelihood function of the distribution parameters represented by L(*θ*|X) = *p*(X|*θ*). The marginal likelihood function represents the marginal distribution of parameter observation data.

(12) $$\begin{array}{c} p\left(X|\alpha \right)=\int p\left(X|\theta \right)*p\left(\theta |\alpha \right)\text{d}\theta . \end{array}$$

Bayesian inference expresses the posterior probability as the product of the likelihood function and the prior probability, namely:

(13) $$\begin{array}{c} p\left(\theta |x,\alpha \right)=\frac{p\left(x|\theta \right)*p\left(\theta |\alpha \right)}{p\left(x|\alpha \right)}\propto p\left(x|\theta \right)p\left(\theta |\alpha \right). \end{array}$$

The mentioned general approximation theory and Bayesian inference theory are regarded as the theoretical basis of deep learning networks.

### 2.3. Multimodal Medical Data

#### 2.3.1. HU Value Processing

For DICOM-type stored CT images, the commonly used Python processing library interface cannot automatically convert the read value to Hu value, so manual conversion is required [24]. For CT images, there is a specific measurement method in the medical field, namely, the Heng's Unit (HU), also known as the CT value. It is a linear mapping of the linear attenuation coefficient of the measured medium, which reflects the degree of absorption of X-rays by the tissue.

(14) $$\begin{array}{c} H=\text{pixel}*S+I. \end{array}$$

The slope represented by S and the intercept represented by I can be read from DICOM format images. It represents the slope and intercept of the conversion. pixel represents the gray value of a pixel.

#### 2.3.2. Histogram Equalization

This article can enhance the overall contrast effect of the image, especially when there is no significant difference in the contrast of the useful part of the image [25]. Histogram equalization is a method of adjusting the contrast using an image histogram. Histogram equalization provides better brightness distribution on the histogram. It improves local contrast without affecting the overall contrast. The specific conversion process is as follows: Calculate the number of times each pixel value in the gray image appears in the gray image.

(15) $$\begin{array}{c} p_{x}\left(n\right)=p\left(x=n\right)\\ =\frac{n_{i}}{n},\;0\leq n<H. \end{array}$$

H is the maximum gray value in the image, *n* is the number of pixels in the image, and *P*(*n*) is the ratio of the number of times the pixel value *n* is displayed in the image to all pixels in the image. Define cumulative distribution function, cumulative normalized histogram, corresponding to Px. The formula is as follows:

(16) $$\begin{array}{c} Cdf_{x}\left(n\right)=\sum_{j=0}^{n}p_{x}\left(j\right). \end{array}$$

Create a mapping transformation formula like *y* = *T*(*x*), and perform a formula transformation on each value in the original grayscale image. The generated *y* cumulative probability function can be linearized in all value ranges for a long time, and the formula is as follows:

(17) $$\begin{array}{c} Cdf_{y}\left(n\right)=iK\text{,} \end{array}$$

where *K* is a constant. According to the nature of CDF:

(18) $$\begin{array}{c} Cdf_{y}\left(y^{\prime }\right)=Cdf_{y}\left(T\left(k\right)\right),\\ =Cdf_{y}\left(k\right), \end{array}$$

where *k* belongs to [0,1], and finally the histogram equalization result can be obtained by the following formula:

(19) $$\begin{array}{c} y^{\prime }=y\left(\max\left\{x\right\}-\min\left\{x\right\}\right)+\min\left\{x\right\}. \end{array}$$

## 3. Experiments on Factors Affecting Neuronal Apoptosis

### 3.1. Extraction of Neuron Signals

The basic unit of the human brain nervous system is the neuron cell, that is, the biological neuron. It is composed of about 10 billion neurons, and each neuron is connected to about 10,000 other neurons [26].  Figure 2 shows the main structure of a single neuron cell, which is composed of cell bodies, axons, and dendrites.

The main difference between nerve cells in the human brain and cells in other parts of the body is that nerve cells can generate, transmit, and process electrical signals. The neuron cell body is divided into inner and outer parts by cell membrane, resulting in different potentials inside and outside the membrane. Normally, the external potential is higher than the internal potential to form the internal and external potential difference, that is, the membrane potential. The membrane potential of neuron cells changes with synapses and the potential changes can be accumulated. That is to say, the membrane potential of the neuron is the sum of the potentials produced by all the synapses connected to it. If the membrane potential gradually rises above a certain threshold, the neuron will produce a neuron pulse, and the number of pulses emitted by the neuron cell when excited is affected by the neuron membrane potential [27]. There is a certain time delay when nerve information is transmitted through synapses, which is generally 0.3ms–1.0 ms for warm-blooded animals.

The neuron firing sequence ISI refers to the time interval between the peak and the peak of the neuron firing pulse. Assuming that a pulse is generated at time *t*, the elements in the sequence of ISIs that define the peak-to-peak interval of adjacent action potentials can be represented in Figure 3.

The map of neuron firing is drawn with the time interval of each spike in the neuron firing sequence as the abscissa, and the next spike time interval as the ordinate. The map can reflect some special recurring neuron firing patterns. In the biological nervous system, there are many different forms of charged ions in neuron cells, and it also has neurotransmitters that transmit electrical and chemical signals. At present, most researches are sodium ion, potassium ion, calcium ion, and so on. These ions are the basis for nerve cells to transmit and process information. Normally, the concentration of sodium and calcium ions in neuron cells is lower than that outside the neuron cell membrane, while the concentration of potassium ions is higher than that outside the neuron cell membrane. At the same time, the neuron cells remain relatively static due to the barrier function of the cell membrane in the static state, and have different permeability to different ions in different states. When the neuron cell membrane is in a static state, the neuron cell membrane is more permeable to potassium ions than sodium ions and calcium ions. Therefore, more positive charges on the neuron cell membrane form an internal and external potential difference [28]. When the movement of internal and external ions reaches a relative balance, a constant potential difference between the inside and outside of the membrane will form, that is, the resting potential.

Figure 4 shows the simulation results of the H-R model of normal and rapid firing of a single neuron. The horizontal axis represents the simulation time, and the vertical axis represents the membrane potential value.

Figure 4 shows the firing model of a single HR neuron, with parameters *r* = 0.0021 and I = 3.024. It can be seen from the simulation results that the discharge model of the HR neuron model is determined by the control parameter *r*. But this parameter is not necessarily the only parameter that controls the model type [29]. From the figure, it can be inferred that when *r* fluctuates in a certain numerical interval, an irregular neuron firing model can be obtained, that is, a rapid firing model. As shown in the figure, after many simulation tests, the interval is [0.0014,0.0091]. According to relevant data, *r* = 0.0021 is selected here. The characteristic of this discharge model is that the discharge appears as a “cluster..

When *r* is greater than 0.0091 and less than a certain value, here we take *r* = 0.022 to obtain a regular neuron firing model. Its characteristic is that each discharge interval is approximately equal, and the sequence interval ISI changes little. From the simulation results, it can be inferred that there is a specific value from the irregular model to the regular model.

By fixing the input current I and changing *r*, the simulation results and ISIs sequence of different control parameters are obtained, as shown in Figure 5:

The upper picture shows the neuron firing pattern, and the lower picture shows the corresponding ISIs sequence scatter diagram. It can be seen from the neuron firing model image that when the value of I is very small, the neuron appears in a chaotic firing state [30]. When I increases, the chaotic state transitions to the discharge state. From the corresponding ISIs sequence scatter image, it can be seen that when I increases, the value of ISI gradually decreases and the frequency gradually increases.

Figure 6 is the time interval sequence ISIs of the regular issuance model, where I = 3.024 and *r* = 0.022. It can be seen from the simulation diagram that a neuron has one impulse every time it fires, and the abscissa indicates the time point when the pulse is obtained. The interval between the two pulses is the ISI, and the pulse distribution is relatively uniform.

Studies have confirmed that the AKT/NF-KB signaling pathway is closely related to epilepsy. AKT plays an important role in cell proliferation, migration, and cell survival, and NF-KB is an important downstream target protein of AKT. MK2206 is a specific allosteric inhibitor of AKT. It can inhibit the phosphorylation of AKT, thereby inhibiting AKT activation. MK2206 can effectively inhibit the proliferation of a variety of malignant tumor cells, promote tumor cell apoptosis, and exhibit good anti-tumor activity [31]. Necroptosis is a new type of cell death discovered in recent years, which is regulated by special death signaling pathways. Receptor interacting proteins 1 and 3 are very important regulatory proteins in the necroptotic signaling pathway.

### 3.2. Establish a Neuron Epileptiform Discharge Model

The experimental subjects were mice, and the experimental group and control group mice were euthanized. Then, hippocampal tissues on both sides of the ice surface were separated after washing with physiological saline, the left and right hippocampus were put into the labeled imported coming cryotubes, and stored in liquid nitrogen tanks. Bilateral hippocampus was used for experiments, the left hippocampus was used to extract total protein, and the right hippocampus was used to extract nuclear and cytoplasmic proteins. Three rats in each group were directly decapitated to take their brains for paraffin sectioning. The brain tissues were placed in 4% paraformaldehyde and immersed for 24 hours for paraffin embedding. Paraffin tissue sections were used for HE staining and NISSLE staining of the hippocampal tissue. The sample size of the experimental pilo90 mg group was 8, the Racine score reached SE5, and the Racine score did not reach SE3. The epilepsy rate was 62%. The sample size of the control pilo90 group was 10, the Racine score reached SE10, and the Racine score did not reach SE0. The epileptic rate was 100%. The sample size of the control pilo30 group was 16 rats, the Racine score reached SE8, and the Racine score did not reach SE8, and the epileptic rate was 50%. Compared with the control pilo90 mg group, the epilepsy rate of the experimental pilo90 mg group was significantly reduced (*p* < 0.05), as shown in Table 1 and Figure 7.

The mice in the experimental group and the two control groups had no obvious abnormal changes after being injected with lithium chloride. Peripheral cholinergic reactions such as erect hair, salivation, eye congestion, etc., began to appear within a few minutes after intraperitoneal injection of pilocarpine, which lasted for about ten minutes. Different degrees of seizures occur simultaneously or sequentially, such as staring, less moving, blinking, chewing, sniffing, and groping. It can be seen that the head and neck are raised and there are tremors repeatedly [32]. The seizures develop further, with nodding tremor, unilateral or bilateral forelimb twitching, and they are in a semi-upright posture. It often leads to spasms of the hind limbs, followed by falling backwards or rotating, and seizures of tonic-clonic all over the body. During the course of the disease, the mice appeared sluggish. After SE lasted for 60 minutes, intraperitoneal injection of diazepam terminated the seizure, and the mice were in a state of inhibition and consumption, with reduced response and activity.

Comparing the experimental pilo90 mg group with the control pilo90 mg, the incubation period was significantly prolonged, *p* = 0.046 < 0.05. Compared with the control pilo90 mg group and the control pilo30 mg group, the incubation period was significantly shortened *p* = 0.002 < 0.01, as shown in Table 2 and Figure 8.

MK2206 has a specific inhibitory effect on AKT and has good safety. At present, its research on tumor diseases has entered the second clinical phase, and there is no research report on MK2206 in epilepsy. This article requires in-depth research, and Mk2206 is expected to become a new method of epilepsy treatment.

Studies have confirmed that the AKT/NF-KB signaling pathway is closely related to epilepsy. MK2206 is a specific allosteric inhibitor of AKT. Due to the excellent efficacy and safety in tumor treatment, it has now entered the second phase of clinical research. Necroptosis is a new method of cell death discovered in recent years, and it has become a research hotspot at present. It has been shown that in most cells, the binding of death receptors and ligands can activate the apoptotic pathway. If caspase is over-activated, the apoptotic pathway is blocked and the cells enter the necrotic pathway, leading to necroptosis. In addition, cells can also cause cell necrosis by triggering pathogen recognition receptors. Such receptor families usually include toll-like receptors, cytoplasmic receptors, and RIG-like receptors. These receptors can recognize the molecular family of bacteria or viruses related to pathogens, such as lipopolysaccharide LPS, flagella, etc., thereby inducing innate immunity and leading to cell death. In addition to the mentioned pathways that mediate necroptosis, researchers have also found that calcium ion concentration, phospholipase, intracellular reactive oxygen species, and calpain can mediate necroptosis. In the process of cell proliferation, excessive DNA damage caused by aerobic stress can lead to excessive activation of RIP1, which leads to cell necrosis [33]. Studies have found that RIP3 can control the balance between apoptosis and necrosis pathways, which means that apoptosis and necrosis can be transformed. In the cell, if the expression level of RIP3 is high, the cell will die. Conversely, if the expression of RIP3 is low, the cells will undergo apoptosis.

### 3.3. Diagnosis of Liver Cirrhosis Based on Deep Learning

In the previous chapter, this article gave a general analysis and overview of the establishment of neuron epileptiform discharge model, and conducted research and verification on the ideas and algorithms involved in each module. In order to consider the accuracy and universality of neuron technology, this paper proposes to use a multi-modal high-precision fusion algorithm for optimization. Based on various performance indicators, this article will also verify the high-precision indoor and outdoor scene recognition technology based on multi-modal fusion in order to achieve better results. Medical imaging is an important tool for the study of clinical diseases. It plays an irreplaceable role in the early screening, treatment and subsequent rehabilitation, detection and management of the disease. However, the traditional artificial medical imaging diagnosis method still has many problems, such as the imbalance between the supply and demand of the doctor and the patient, and the heavy burden of the hospital staff. Medical imaging diagnosis is highly subjective and requires high experience. With the rapid development of deep learning in the image field, many deep learning methods have gradually been used in the processing and analysis of medical images in recent years to assist doctors in automatic diagnosis and improve work efficiency. However, considering the complexity of medical recognition tasks and the small sample size of medical images, the current mainstream research is monomodal imaging research, which still has some shortcomings. Because single-modal images are often unable to comprehensively and accurately express relevant pathological information, multiple images of different modalities can reflect the relevant information of the lesion from different aspects, making up for the lack of data and the disadvantages of a single information perspective. Therefore, based on multi-modal image data, the use of deep learning for early disease screening is of great significance for improving the accuracy of medical task recognition and assisting doctors in decision-making and diagnosis [34, 35]. This article focuses on the research of multi-modal medical imaging, and mainly conducts two groups of disease classification experiments based on multi-modal medical imaging.

The network model is pretrained through the large-scale data associated with the sample set to obtain the initialization parameters. Its effectiveness is that the network model is multi-level when learning sample features. And, the level is different; its characteristic expression is also different. With the deepening of the level, the greater is the difference of the learned sample information. In the lower level, the characteristics of the image described are less different, such as the color, contour, shape, size, and edge. The sample set image has a certain similarity and relevance to the pretrained sample set image. So, these low-level parameters can be shared. This article uses MNIST natural images. The dogs and cats in the data set are used as pretraining samples, as shown in Figure 9.

In deep learning, the deeper the model, the more neural nodes, and a larger sample set is needed to optimize many parameters of the model. If the sample set is small, each parameter cannot be trained to the best, and it is very easy to produce over-fitting. The research in this article is the image recognition of liver pathology in the medical field. The number of sample sets is far less than that of the natural image sets in life. In the transfer learning method, the natural image set by MNIST is used as the starting domain of Di, and one thousand classifications are used as the learning task Ti. After pretraining, the model parameters are retained, and then the model is applied to the medical liver pathology images in this paper for training. Finally, it improves the pan-China capability of the model and effectively prevents over-fitting. Many methods and applications have also confirmed its advantages [36]. The current transfer learning methods are mainly concentrated in two aspects: one is to keep the learned parameters unchanged and use them directly, and the other is to fine-tune the learned parameters.

Based on the explanation, this article established the SqueezeNet convolutional neural network model. The 1.2 million images in the ImageNet dataset have undergone thousands of classification trainings to obtain a pretrained classification model. The model parameters are shown in Table 3.

This article selects 1500 pathological images of the liver. Among them, 1,000 are used as the training sample set (600 are normal livers, 400 are affected by cirrhosis), and 500 are test samples (300 are normal livers and 200 are affected by cirrhosis). The experimental environment is the Linux system, Intel i5CPU, running memory 8G, running using caffe framework. This article adopts the second transfer learning method, fine-tuning training, using natural image sets for pretraining, and applying the obtained parameters to medical images to fine-tune the parameters. As shown in the comparison in Figure 10, this will further improve performance and increase the recognition rate of the original image. The recognition rate is increased from 67.2% to 84.5%, and the time will be reduced. This proves the effectiveness of transfer learning.

This article adds typical deep learning models such as AlexNet, GoogleNet, and LeNet for comparison. After reducing the model size to verify the performance of the lightweight convolutional neural network structure SqueezeNet with fewer parameters, the comparison results are shown in Table 4.

The model can distinguish each liver pathology image and give the probability of the class each pathology sample belongs to [37]. For example, the result of the first medical pathological image of liver cirrhosis is that 99.4% belong to cirrhosis, and 0.5% belongs to normal liver. And, the judgment given by the fourth normal liver sample model is that 99.5% are normal livers and 0.5% is diseased. It can be seen that it is very important and helpful for the practical application of clinical medical diagnosis, and it can help physicians to identify which disease the pathological image belongs to. The physician can also refer to the probability results given by the model. Because this article only trains patients with liver cirrhosis, the results will only show the probability of normal disease and liver cirrhosis. If a variety of liver diseases can also be trained and applied, after completing the training, it will give the probability of each disease.

## 4. Discussion

Although this article has made some progress on the basis of other scholars' research, the content of this thesis is not perfect due to time constraints. The follow-up research can be carried out in the following contents: This article studies the firing pattern, coding, and parameters of HR neurons. Follow-up can be combined with another research topic on synapses to form a neural network circuit composed of HR neurons to simulate the algorithm and performance of the neural network. This paper only studies the synchronization of 3 and 4 neurons in the fully connected network and the synchronization of 4 neurons in the star network and the nearest neighbor connection network. Later, the number of neurons can be increased, and the synchronization problem of larger-scale neuron networks can be studied.

## 5. Conclusion

This article mainly studies the neuron model's firing pattern and the influence of parameters on the pattern and neuron information coding. As for the research of the neuron model, domestic and foreign research is in the exploratory stage, so the research has certain difficulty. Although there are some related neuron models, and most of these models are based on physiology. It is difficult to realize large-scale neural network networking. The content and results of this thesis are just basic work for further research on neural networks. This article adopts the method of multi-modal fusion deep learning, fine-tuning the training; the neuron recognition rate is increased from 67.2% to 84.5%%, and the time is also reduced, which proves the effectiveness of deep learning.

## Figures and Tables

**Figure 1:** Linear weighted fusion structure diagram.

**Figure 2:** Neuron structure.

**Figure 3:** Diagram of ISIs sequence calculation.

**Figure 4:** (a) Rapid firing model and (b) regular firing model.

**Figure 5:** Neuron firing model and ISIs sequence diagram (*r* = 0.0021).

**Figure 6:** Regular discharge pattern and its time interval sequence ISIs.

**Figure 7:** Comparison of epilepsy rate between pilo90 in the experimental group and pilo90 in the control group: *p* = 0.017 < 0.05.

**Figure 8:** The incubation period of pilo90 in the experimental group compared with the pilo90 in the control group.

**Figure 9:** Schematic diagram of transfer learning.

**Figure 10:** Comparison curve of transfer learning (the left picture shows the method after transfer learning).

**Table 1:** Comparison of epilepsy rate between the experimental group and control group.

	Racine score reached SE	Racine score does not reach SE	Sample size	Epilepsy rate (%)
Experimental group pilo 90 mg	5	3	8	62.50
Control group pilo 90 mg	10	0	10	100.00
Control group pilo 30 mg	8	8	16	50.00

**Table 2:** SE latency results of each group (mean ± SEM).

Group	SE latency (min)
Experimental group pilo 90 mg	11.577 ± 1.295
Control group pilo 90 mg	8.239 ± 1.563
Control group pilo 30 mg	5.689 ± 2.756

The incubation period of the experimental pilo90 mg group was significantly longer than that of the control group pilo90 mg

**Table 3:** Squeeze model parameter table.

Parameter\Structure	fire2	fire3	fire4	fire5	fire6
S1∗1	48	16	16	64	16
E1∗1	16	16	64	16	16
E2∗2	48	16	64	16	16

**Table 4:** Comparison table of typical deep learning models.

Experiment	Method	Accuracy (%)	Test time (s)
1	AlexNex	75.57	53
2	SqueezeNet	71.69	41
3	GoogleNet(V2)	60.96	54
4	SqueezeNet + TL	80.64	46
5	SqueezeNet + TL + C-SVM	73.99	55

## Data Availability

The data that support the findings of this study are available from the corresponding author upon reasonable request.
